RETRACTED

# A Critical Scrutiny on Liposomal Nanoparticles Drug Carriers as Modelled by Topotecan Encapsulation and Release in Treating Cancer

**DOI:** 10.1155/2022/7702512

**Published:** 2022-08-09

**Authors:** Hilla Mills, Ronald Acquah, Nova Tang, Luke Cheung, Susanne Klenk, Ronald Glassen, Magali Pirson, Alain Albert, Duong Trinh Hoang, Thang Nguyen Van

**Affiliations:** ^1^Department of Medical Science, University for Development, Accra, Ghana; ^2^RD Lab, The Hospital Institute for Hebal Research, Toluca, MEX 50200, Mexico; ^3^Research Institution of Clinical Biomedicine, Hospital University Medical Centre, Ulm 89000, Germany; ^4^Industrial Research Group, International College of Science and Technology, Route de Lennik 800, CP 590, Brussels 1070, Belgium; ^5^Clinical Analysis Lab, Center of Bio-Medicine, Hanoi, Vietnam

## Abstract

The medical field is looking for drugs and/or ways of delivering drugs without harming patients. A number of severe drug side effects are reported, such as acute kidney injury (AKI), hepatotoxicity, skin rash, and so on. Nanomedicine has come to the rescue. Liposomal nanoparticles have shown great potential in loading drugs, and delivering drugs to specific targeted sites, hence achieving a needed bioavailability and steady state concentration, which is achieved by a controlled drug release ability by the nanoparticles. The liposomal nanoparticles can be conjugated to cancer receptor tags that give the anticancer-loaded nanoparticles specificity to deliver anticancer agents only at cancerous sites, hence circumventing destruction of normal cells. Also, the particles are biocompatible. The drugs are shielded by attack from the liver and other cytochrome P450 enzymes before reaching the desired sites. The challenge, however, is that the drug release is slow by these nanoparticles on their own. Scientists then came up with several ways to enhance drug release. Magnetic fields, UV light, infrared light, and so on are amongst the enhancers used by scientists to potentiate drug release from nanoparticles. In this paper, synthesis of liposomal nanoparticle formulations (liposomal-quantum dots (L-QDs), liposomal-quantum dots loaded with topotecan (L-QD-TPT)) and their analysis (cytotoxicity, drug internalization, loading efficiency, drug release rate, and the uptake of the drug and nanoparticles by the HeLa cells) are discussed.

## 1. Introduction

Drugs were invented to treat a plethora of diseases. However, the drugs pose some undesired effects. In the case of chemotherapy, normal cells are damaged because the drugs do not specifically hit the cancer cells [1]. Consequently, the doses are limited (the therapeutic window is the primarily targeted dose). Chronic chemotherapy might coerce cancer cells to resist the anticancer agents, which is very common [2, 3]. Drug efficacy has to be achieved; otherwise, toxicity is inevitable in the event that drug concentration overshoots the therapeutic window [4]. The human body itself has barriers that serve to protect the system from intrusion by poisonous substances. Amongst such barriers is the blood-brain barrier (BBB), which makes it difficult to treat neurodegenerative diseases [5]. Drugs are considered foreign and are thus subject to expulsion. The cytochrome P40 enzymes, glutathione, the liver, kidney, and many other biological molecules like P-glycoproteins are responsible for xenon compound expulsion. These affect drug bioavailability (F), and reaching a steady-state concentration is daunting [6].

RETRACTED

According to Du et al. [4], nano drug carriers have been shown to greatly counteract the highlighted challenges. It is reported that a number of endogenous and exogenous drug carriers are under scrutiny. Endogenous drug carriers like exosomes and cell membranes are being studied [7, 8]. Exogenous drug carriers such as nanoparticles [9], dendrimers [10], starch microspheres, ethyl cellulose microspheres, albumin microspheres, gelatin microspheres [11, 12], and liposomes [13].

Figure 1 shows some of the liposomal nanoparticle enhancers, among others. Nano delivery systems mitigate toxicity while improving bioavailability. It is reported that liposomes are characterized by biodegradability, biocompatibility, and low toxicity [14–16]. The liposomes can be modified by enveloping them with stable polymers such as oligosaccharides, polysaccharides, glycoproteins, and synthetic polymers with the intention of increasing their half-lives [17]. A controlled process can be used to synthesize liposomes that are capable of carrying either water-soluble or fat-soluble drugs. Such drug carriers are of the magnitude of 100–150 nm. The modified liposomes stealth phagocytosis of the reticuloendothelial system during circulation in the blood, thus toxicity is reduced [18]. It was observed that liposomes, based on the retention effect and tumor enhanced permeability, can accumulate at the cancer site, thus improving drug efficacy [19–21]. Notwithstanding, the rate at which the liposomes release drugs is relatively slow. As a result, a number of response triggers have been studied that enhance drug release. Examples of such response triggers are temperature [22], microwave [23], photodynamic conversion [24], pH [25], and ultrasound [4, 26].

## 2. Topotecan

Figure 2 shows the structure of the topotecan. Topotecan is a hydrophilic anticancer drug that is semisynthetic. It is known that TPT is derived from camptothecin. The drug works by interfering with the protein topoisomerase 1. The drug specifically affects the Topo-1 DNA, forming a ternary complex known as the ‘‘drug-Topo1-DNA” complex [4]. The FDA approved the use of TPT for treating small cell lung cancer and ovarian cancer. It is reported that TPT has a broad spectrum of anticancer activities (i.e., it kills a variety of tumors). One of the major disadvantages of the drug under physiological conditions is that the ring opening of the drug structure results in ineffectiveness, thus affecting drug efficacy [27, 28]. To circumvent the aforementioned drawback, Tarhan et al. [29] prepared special nanoparticles, which were referred to as magnetic dextran nanoparticles branched with N*α*N*α*-Bis (carboxymethyl)-L-lysine hydrate. Seleci et al. [30] prepared a variety of lipid nanoparticles, including LQ-Dots, which were loaded with TPT.

RETRACTED

This review article serves to highlight the theragnostic role played by liposomes in drug delivery systems, enhancing drug bioavailability and efficacy while lowering drug toxicity. In this paper, a very close investigation of the preparation of TPT-loaded quantum dots and the use of liposomes in cancer treatment is carried out.  Table 1 shows some of the lipid-encapsulated drugs approved by the FDA.

### 2.1. Liposome-Nanoparticle Hybrids

Seleci et al. [30] acknowledged that nanomedicine is a multifunctional discipline. The team probed the preparation, characterization, and *in vitro* evaluation of theragnostic liposomes. The team used topotecan (TPT), a hydrophilic drug analogous to camptothecin, as a model drug. The Quantum dots (QDs) are exceptional promising nanoparticles characterized by fluorescent properties such as high photochemical stability, narrow emission spectra, broad absorption spectra, high quantum yields, and resistance to photobleaching [32–34]. Owing to these properties, QDs have been studied for biochemical applications as fluorescent probes. It is reported that QDs are particularly useful for *in vivo* cell labeling and imaging [35–38].  Table 2 shows some of the applications of nanoparticles (NPs) in the medical field.

### 2.2. Preparation of Liposome-QD Hybrids

A number of modifications are made with the intention of surmounting the aforementioned drawbacks. It is reported that a broad spectrum can improve QDs [39]. Notwithstanding, surface modifications decrease fluorescence photostability and intensity [30, 40].

According to Muthu et al. [41], LQD exhibited excellent potential. It is reported that Tian et al. loaded with LQD [42]. In addition, in one study, L-QDs loaded with apomorphine were investigated for bioimaging and brain targeting. It was observed that the liposomes accumulated in the brain to a large extent [43]. Moreover, Muthu et al. tailor-made the folic acid-conjugated theragnostic liposomes purporting to carry out the targeted co-delivery of quantum dots and docetaxel [30, 41].

RETRACTED

### 2.3. Methodologies

Reference [30] used the thin film hydration method to synthesize L-QD hybrids [44]. In a round-bottomed flak that contained chloroform (an organic solvent) [45].

### 2.4. TPT Encapsulation

The drug (TPT) was loaded into the L-QD vesicles using a pH-gradient technique [46]. The lipid-QD dried thin film obtained, things can be determined by a ratio of drug weight encapsulated to the initial drug weight before encapsulation.

(1) $$\begin{array}{c} \%\text{ EE}=\frac{W\text{en}}{W\text{ total}}\times 100. \end{array}$$

The above equation was used to calculate encapsulation efficiency, where *W*_en_ is the drug weight encapsulated in the L-QDs and *W*_total_ is the initial drug weight [47]. Encapsulation efficiency was determined following L-QD-TPT hybrid vesicles lysis by diluting purified liposomes in acidic methanol (1% trifluoroacetic acid in methanol). Known concentrations of free TPT were used for curve calibrations by measuring fluorescence emission at 530 nm using a fluorospectrometer (NanoDrop 3300, Thermo Fisher Scientific Inc., Waltham, MA, USA).

Formulation fluorescence spectra were determined by a spectrofluorometer while an Olympus BX41 fluorescence microscope was used to capture TPT and QD localizations in a big liposome. Zetasizer Nano-ZS (Malvern Instruments, Malvern, UK) was used to analyze the zeta potential (*ζ*) and particle size distribution of the liposomes. A parameter known as the polydispersity index (PDI) was reported as the size distribution width. In their study, the samples were diluted using a 1 : 100 (*v*/*v*) ratio with ddH_2_O. These diluted samples were first equilibrated for 3 minutes prior to measurements. At room temperature, measurements were taken in triplicates. The team tested and examined the stability of the samples (liposomal formulations) by storing them [30].

### 2.5. *In Vitro* Drug Release Assay

Reference [30] carried out a drug release experiment using the dialysis technique. The team prepared the LQD. The release medium was replenished by the same amount of fresh buffer. A calibration curve was used to quantify the TPT released. The concentrations were studied at 530 nm using a spectrofluorometer.

### 2.6. Cell Culture

Reference [30] cultured it. In a medium that contained 1.0% penicillin/streptomycin (P/S) and 10% fetal calf serum (FCS), cells were grown. The medium conditions were 5.0% CO_2_ and 37°C.

RETRACTED

### 2.7. Cytotoxicity Assay

Cytotoxicity of liposome formulations was carried out using the MTT (3-(4, 5-dimethylthiazol-2-yl)-2, 5-diphenyltetrazolium bromide) assay. In a 96-well tissue plate (Sarstedt, Newton, MA, USA), 8 × 10^3^ cells were seeded in a volume of 200 *µ*l and then grown for 72 hours. Cells produced a formazan complex during the incubation period. Purple-colored salts were removed from the cells. Then UV-Vis absorption was measured using a reference wavelength in the range of 570–630 nm [30].

### 2.8. Cellular Uptake

The cellular uptake of liposomal formulations and TPT by HeLa cells was studied through flow cytometry. Cells (5 × 10^5^) were collected, incubated with the samples for 2 h, and then washed twice with PBS. Flowing Software 2 was used to analyze dot plot and histogram data [30].

## 3. Discussion

Focusing on the study conducted by Seleci et al. [30], the liposomes were formulated using distearoylphosphatidylcholine (DSPC) and cholesterol in the ratio of 7 : 3 respectively. The team wanted membrane rigidity and thus chose DSPC over any other possible phospholipids like dimyristoylphosphatidylcholine (DMPC) and egg phosphatidylcholine (EPC). The DMPC increases liposomal drug retention [48, 49]. It was observed that sufficient cholesterol (≤30%) prevented leakage of encapsulated contents by decreasing contents' solubility and increasing contents' stability [50, 51]. It is reported that cholesterol could also enhance membrane hydrophobicity [52]. Seleci et al. [30] chose the simple and commonly used method of liposomal synthesis, which is a thin layer hydration. The pH technique works on the basis that a pH gradient is a driving force that accumulates weakly basic molecules in acidic vesicles. TPT was loaded using this approach, and its active lactone form was retained till release. Liposomal and free drug fluorescence spectra revealed both TPT and QD peaks simultaneously, thus confirming the coexistence of the two in the vesicles. The team carried out molecules' fluorescence localizations in a large liposome.

It is emphasized that the nanoparticles' physicochemical properties are crucial in protein interactions [53]. Piling evidence supports those nanoparticles in magnitude. There are some other studies [54, 55]. In this regard, Seleci et al. [30] determined liposomes' surface charge and hydrodynamic parameters by carrying out Dynamic Light Scattering (DLS) and *ζ*-potential analysis. The average size of the plain liposomes was found to be 132 nm. An increase in liposome size by 6 nm was detected following entrapping the QD in the lipid bilayer. This could only be explained by the successful encapsulation of molecules. Encapsulation of the TPT did not alter the size of the L-QD. The researchers examined liposomal stability upon storage. The observations were that at 4°C in a space of over 2 months, there were no significant changes in *ζ*-potential, size distribution, and polydispersity index (PDI).

RETRACTED

According to Deng et al. [56] and Gessner et al. [57], the higher surface charge of nanoparticles has effects on the amount of protein adsorption.

Protein corona composition on the surface. A number of studies revealed the mechanism [58–61]. In the study conducted by Seleci et al. [30], efficiency was found to be approximately 40%. The QD integration was found to have affected it. Furthermore, the hybrid liposomes had better physicochemical properties.

An important aspect of treatment, drug release, was analyzed *in vitro* by Seleci et al. [30]. The team came up with an L-QD-TPT drug release profile following its determination using the dialysis method, which is the most common approach for nanoparticle drug release analysis. The researchers created an environment that mimics normal human tissue conditions with a pH of 7.4 and a tumor microenvironment (pH 5.6) at a temperature of 37°C. It was observed that TPT release was higher in an acidic environment as compared to a neutral one. In the first 4 hours, the drug release was rapid due to the modest initial burst of the L-QD-TPT nanoparticles, with the acidic-environment nanoparticles reaching about 33% cumulative drug release while neutral-environment nanoparticles scored 25%. Slower rate release occurrs for up to 32 hours. Thereafter, TPT release rates were observed to be 39 and 45% for the neutral and acidic conditions, respectively. Higher cumulative drug release in acidic conditions is attributed to the protonation of TPT, hence increasing its solubility [61].

Seleci et al. [30] observed that cells treated with samples (TPT, L-QD, L-TPT, and L-QD-TPT) had higher fluorescence signals as compared to control cells, which were not subjected to samples. The observed fluorescence signal measurements for TPT, L-TPT, and L-QD-TPT were 2472 a.u., 3839 a.u., and 4007 a.u., respectively. The discrepancies in fluorescence signal measurements are explained by different mechanisms by which HeLa cells take in the formulations. It is reported that free TPT enters the cells and makes its way into the cells via endocytosis [62, 63].

Seleci et al. [30] examined the L-QD-TPT-treated cells by fluorescence microscopy. The fluorescent model drug (TPT) was found unsurprising in the nuclei of the cells since it is a topoisomerase-I inhibitor, to execute its toxicity [64, 65]. In their study, the blue and green fluorescence from 4′, 6-diamidino-2-phenylindole (DAPI), and TPT, respectively, matched very well. The DAPI was used to stain the nuclei of the cells.

RETRACTED

Furthermore, the researchers determined the cytotoxicity of TPT and free liposomal formulations on HeLa cells using a 3-(4, 5-Dimethylthiazol-2-yl)-2, 5 diphenyltetrazolium bromide (MTT) assay. The assay works based on the principle that only viable cells with active metabolism convert MMT into formazan, a purple-colored substance. The quantification of formazan is carried out by taking absorbance readings at 570–630 nm reference wavelengths. Seleci et al. [30] found out that L-QD caused no cytotoxicity. The reason is that the lipid bilayer shielded the cells from harm effectively. The same results were reported by Chinnathambi and colleagues. In their study, phosphoethanolamine (polyethylene glycol)-based phospholipid micelles were used to envelope CdSe/ZnS QDs. The QDs in the concentration range of 0–25 *µ*g/ml almost showed no toxicity in A546 and HeLa cell lines following 24 hour-exposure. However, in the case of Seleci and colleagues, L-QD-TPT and L-TPT obviously posed toxicity on HeLa cells after 24 hour-exposure. This is due to high L-QD-TPT and L-TPT intake by the cells, and the TPT concentration delivered was obviously higher than that of free TPT. It is reported that the same results were obtained by Hao and colleagues [66].

Versions of the liposomal nanoparticles exist. These include magnetic nanoparticles [67]; thermosensitive liposome-in-gel [5]; transferrin receptor (TR)-targeted liposomal cisplatin [68]; magnetic thermosensitive cationic liposomes [69] and so on. Novel technologies have also been reported [70, 71].

## 4. Conclusion

Liposomal nanoparticles increase drug bioavailability while lowering drug toxicity. Controlled drug release is also achieved and is an important aspect of treatment where steady-state concentrations are maintained, hence drug efficacy is achieved. Therefore, nanomedicine is improving the diagnosis and treatment of patients tremendously. In this paper, the synthesis of liposomal nanoparticle formulations (liposomal-quantum dots (L-QDs), liposomal-quantum dots loaded with topotecan (L-QD-TPT)) and their analysis (cytotoxicity, drug internalization, loading efficiency, drug release rate, and the uptake of the drug and nanoparticles by the HeLa cells) were discussed.

## Figures and Tables

**Figure 1:** Some of the liposomal nanoparticle enhancers, among others.

**Figure 2:** The structure of topotecan.

**Table 1:** Some of the lipid-encapsuled drugs approved by the FDA [31].

Drug	Date of first approval	The drug treats:	Company
Doxil	1995	Kaposi's sarcoma, ovarian cancer, multiple myeloma	Janssen
DaunoXome	1996	Kaposi's sarcoma	Galen
Marqibo	2012	Acute lymphoblastic leukaemia	Acrotech
			Biopharma
Onivyde	2015	Metastatic pancreatic cancer	Ipsen
Vyxeos	2017	Acute myeloid leukaemia	Jazz
			Pharmaceuticals
Onpattro	2018	Transthyretin-mediated amyloidosis	Alnylam
			Pharmaceuticals

RETRACTED

**Table 2:** Some of the applications of nanoparticles (NPs) in the medical field [31].

Application	Description
Genome editing	NPs carry CRISPR components to the nucleus
Stratification of patients basing on genetic information and biomarkers	Antibody-targeted NPs reach cancer cell with complementary receptors
Modulation of the immune system and response	NPs deliver mRNA vaccines in the system
Determination of pharmacokinetics changed by disease states	NP-based imaging unveils levels of enhanced permeation and retention (EPR).
Autologous cell therapies creation	NPs generate chimeric antigenic receptor (CAR) T cells for cancer immunotherapy

## Data Availability

The data used to support the findings of this study are included within the article.
